RETRACTED

# Intelligent Assessment of Mental Health Based on Multisource Information Fusion

**DOI:** 10.1155/2022/7149817

**Published:** 2022-01-27

**Authors:** Yumei Jing

**Affiliations:** Mental Health Education and Counseling Center, Hubei Normal University, Huangshi 435000, China

## Abstract

Mental health problems will seriously damage social harmony and family happiness. This paper proposes a study on mental health intelligence assessment based on multisource information fusion. Combining the data description of UPI and SCL-90 and the corresponding task requirement analysis, the multisource information fusion visualization based on the Circos diagram is designed and realized, and the parallel coordinate visualization is established. The MDS algorithm is used to project multidimensional survey objects into low-dimensional visualization space, and the actual UPI and SCL-90 questionnaire data for 278 students of a certain major at a university provided by the cooperative unit are used. The results show that the mental health problems of student A are serious, and the symptoms of depression and schizophrenia are prominent, so it is necessary to seek psychological experts for corresponding treatment in time. By contrast, student B's mental health problems are also serious, and the user judges that student B still needs further diagnosis and treatment. The correlation analysis results of multisource information fusion are roughly the same as the actual situation, which is convincing. Therefore, the multisource mental health information fusion of college students has a certain correlation and complementarity.

## 1. Introduction

Traditional mental health assessment, especially large-scale mental health assessment, mostly adopts the questionnaire survey method based on a self-rating scale [1]. This method is not timely, and the current psychological state of the subjects who fill in the self-rating scale has a great influence, and its invasive characteristics will also cause the resistance of the subjects and increase the false alarm rate. On the issue of automatic assessment of mental health, the research of this kind of problem mainly discusses the relationship between users' mental health status and their behaviors on online forums or other social networking platforms, and studies whether individuals' mental health can be predicted by their behaviors on online forums or social networking platforms [2]. Although the machine learning method based on the combination of deep learning method and feature engineering and traditional feature engineering performs well, there are still some features that may be neglected. Combining with the deep learning method, the traditional feature engineering method is introduced. To solve this research problem, Meng, Chen, and others found a method compared with the normal control group. Among the poems published by poets who have committed suicide, first-person singular and death-related words are frequently used [3]. Fu, Wang, et al. first manually marked some suicide words as a seed dictionary, and then extended the suicide dictionary based on the similarity between Word2Vec words by training the Word2Vec model [4]. Chen, S. uses the semantic information in HowNet to guide deep online learning of deeper word semantic information to expand the LIWC dictionary, and achieved good results [5]. On the basis of current research, this paper puts forward the research of mental health intelligence assessment based on multisource information fusion, combining the data description of UPI and SCL-90 and the corresponding task demand analysis. Design and realize multisource information fusion visualization based on the Circos diagram, establish parallel coordinate visualization, use the MDS algorithm to project multidimensional survey objects into low-dimensional visualization space, and use the actual UPI and SCL-90 information fusion data provided by the cooperative unit for 278 students of a certain major at a university. Multisource mental health information fusion of college students has certain correlation and complementarity.

RETRACTED

## 2. Method

### 2.1. Data Introduction

UPI and SCL-90 are common forms of information fusion, which are widely used in the investigation and analysis of college students' mental health [6]. UPI data consists of three parts: (1) Basic information of students, including students' individual natural attributes, personal and family history, professional satisfaction, and so on. (2) Questionnaire, including 60 questions, except for 4 false test questions. The remaining 56 topics reflect students' physical and mental health from different angles, including anxiety, distress, depression, interpersonal sensitivity, conflicts, and so on. (3) Auxiliary proposition: it helps psychologists understand and diagnose students' mental health status through students' opinions on specific issues. The SCL-90 is a famous mental health test scale, which includes 90 self-assessment items. The specific evaluation angle includes 10 factors which are somatization, obsessive-compulsive symptoms, interpersonal sensitivity, depression, anxiety, hostility, terror, paranoia, psychosis, and others [7]. According to the distribution of the symptom index, we can effectively identify the mental health status of the respondents; that is, the higher the score, the more serious the corresponding symptoms. For example, the score is 1.0–1.5. It shows that the respondents are psychologically healthy and have no symptoms listed on the scale; a score of 4.5–5.0 indicates that the frequency and intensity of symptoms are very serious [8]. This paper verifies that the data of the visual analysis system comes from the real information fusion data of UPI and SCL-90 accepted by 278 college students in a certain university in the same period. The data includes the basic information of all students, the answers of UPI and SCL-90 questionnaires, the scores of four mental health categories of UPI data, and the scores of nine factors of SCL-90 data.

RETRACTED

### 2.2. System Overview

Combined with the data description of UPI and SCL-90 and the corresponding task demand analysis, this paper intends to provide a visual analysis system tool that can effectively analyze and explore multisource college students' mental health data for college mental health consulting institutions. Firstly, the system imports multisource data of mental health information fusion of college students, including the basic information of 278 students and the answers of UPI and SCL-90 questionnaires. After successfully loading data, the system mainly provides the following visual analysis functions: visualization of multisource questionnaire data of respondents based on the Circos graph, in which a fan-shaped distribution describes the problems in the questionnaire, and color and line chart describe the degree of symptoms, which visually presents the mental health status of respondents.

### 2.3. Multisource Information Questionnaire Fusion Visualization

The traditional mental health questionnaire system pays attention to data collection, but there are limitations in data management and analysis. It usually requires users to export data, use classic statistical software for analysis, and repeatedly load and process data. The process is cumbersome and time-consuming, and the analysis results are uncertain. Furthermore, multisource information fusion usually has different structural descriptions. It is often difficult to effectively explore and analyze the mental health of college students comprehensively and deeply [9]. In order to comprehensively consider multisource information fusion data information, multisource information fusion visualization is designed and realized based on the Circos diagram. The scheme design is shown in Figure 1.

### 2.4. Multisource Information Questionnaire Angle-Related Visualization

There are differences in the overall goal of judging college students' physical and mental health due to the different degrees of detail of the two questionnaires. Therefore, the angle-dependent visualization method of multisource information fusion is designed [10]. The main steps of quickly and intuitively presenting the correlation of information fusion from different analysis angles are as follows:

RETRACTED

#### 2.4.1. Parallel Coordinate Visualization

In order to visually display the characteristic information of multidimensional survey angle of multisource information fusion data, according to 14 angle attribute categories of the two types of questionnaires UPI and SCL-90, a parallel coordinate system is constructed, and each axis corresponds to an attribute category. Then, the total scores of questions obtained by the survey object in each attribute category are calculated, and the scores are mapped to the corresponding coordinate axes and plotted into curves. Furthermore, the overall distribution of survey objects and related characteristics of different survey angles can be intuitively presented through data distribution.

#### 2.4.2. Correlation Coefficient Calculation

In order to further quantify the correlation characteristics between survey angles, the correlation coefficient was introduced to measure the correlation between any two attribute axes in the parallel coordinate system [11]. First, *y*_*iq*_ was recorded as the total score of the question obtained by the survey object *q* in the attribute category *J*, and then the mean score ${\bar{y}}_{i}$ of the survey object in each attribute category was calculated as follows:

(1) $$\begin{array}{c} \rho \left(i,j\right)=\frac{Cov\left(i,j\right)}{\sigma_{i}*\sigma_{j}}. \end{array}$$

(2) $$\begin{array}{c} \frac{\text{Cov}\left(i,j\right)}{\sigma_{i}*\sigma_{j}}=\frac{1}{n-1}\sum_{q=1}^{n}\left(\frac{y_{iq}-{\bar{y}}_{i}}{\sigma_{i}}\right)\left(\frac{y_{jq}-{\bar{y}}_{j}}{\sigma_{j}}\right). \end{array}$$

Among them, I and *J* represent different attribute categories, respectively; N indicates the total number of respondents; *σ*_*i*_ and *σ*_*j*_ represent the standard deviation of object data of different attribute categories; Cov(*i*, *j*) is the covariance between these two attribute variables, and its calculation formula is as follows:

(3) $$\begin{array}{c} Cov\left(i,j\right)=\frac{1}{n-1}\sum_{q=1}^{n}\left(y_{iq}-{\bar{y}}_{i}\right)\left(y_{jq}-{\bar{y}}_{j}\right). \end{array}$$

### 2.5. Multisource Information Uncertainty Visualization

According to the basic data of SCL-90 and UPI2 information fusion, the MDS algorithm is used to project multidimensional survey objects into the low-dimensional visualization space, and the distance difference between the survey objects in the high-dimensional space and the low-dimensional space is kept as consistent or similar as possible [12]. The main steps are as follows:

RETRACTED

#### 2.5.1. Similarity Matrix Calculation

According to the basic information of respondents' answers to questionnaires, count the number of questions with the same answers and measure the similarity of respondents. For example, if two students' questionnaire answers are basically the same, they are considered to have a similar mental health status. Therefore, the similarity matrix of the respondents was obtained according to the questionnaire answer statistics [13].

(4) $$\begin{array}{c} D=\left\{\begin{array}{c} d_{11}...d_{1m}\\ ...d_{ij}...\\ d_{m1}...d_{mm} \end{array}\right\}. \end{array}$$

Among them, *m* represents the number of students who participated in the questionnaire; *d*_*ij*_ indicates the number of questions with different answers in the questionnaires of student I and student *J*.

#### 2.5.2. Dimension Reduction Projection

In order to further visually present the mental health status of the respondents, the MDS algorithm is used to reduce the dimension projection of the multidimensional respondents, that is, the original multidimensional data is projected into the K-dimensional space. *Z* ∈ *R*^*m*×*k*^ is the medium. *z*_*i*_ and *z*_*j*_ represent the coordinates of student I and student *J* in the projection coordinate system.

(5) $$\begin{array}{c} d_{ij}^{2}={\left\|z_{i}-z_{j}\right\|}^{2}. \end{array}$$

(6) $$\begin{array}{c} {\left\|z_{i}-z_{j}\right\|}^{2}={\left\|z_{j}\right\|}^{2}+{\left\|z_{j}\right\|}^{2}-2z_{i}^{T}z_{j}. \end{array}$$

It is assumed that the data objects in low-dimensional space are centralized, ∑_*i*=1_^*m*^*z*_*i*_=0. Furthermore, the left and right sides of formulas (5) and (6) are summed, and the inner product matrix is defined by*B*=*ZZ*^*T*^ ∈ *R*^*m*×*m*^, namely, *b*_*ij*_=*z*_*i*_^*T*^*z*_*j*_. The results are as follows:

(7) $$\begin{array}{c} b_{ij}=-\frac{1}{2}\left(\frac{1}{N^{2}}\sum_{i=1}^{N}\sum_{j=1}^{N}d_{ij}^{2}-\frac{1}{N}\sum_{j=1}^{N}d_{ij}^{2}+d_{ij}^{2}\right). \end{array}$$

Using formula (7) to decompose matrix B, the projection *Z* of the original multidimensional data object in k-dimensional space is finally obtained.

#### 2.5.3. Participation *F*^3^*TMH*_−_*V* Voting Model Generation Algorithm

Input: training data set *D*, candidate feature set *ψ*. The results show that they include behavior attribute feature BAF, language feature LGF, n-grams feature NGF, topic feature TPF, and word vector feature WEF.

Output: participation *F*^3^*TMH*_−_*V* voting models, such as formulas.

(8) $$\begin{array}{c} f=\arg\max F_{1}\left(m\left(f^{\prime }\right)\right),\varepsilon =\underset{f^{\prime }\in \psi }{\max F_{1}}\left(m\left(f^{\prime }\right)\right). \end{array}$$

The single feature that makes the model performance optimal and the threshold value of the voting model performance are found.

(9) $$\begin{array}{c} G=\left\{f\right\},M=\left\{m\left(f\right)\right\},\psi =\psi -\left\{f\right\}. \end{array}$$

(10) $$\begin{array}{c} {\text{WHILE}}_{\psi }\neq \varphi . \end{array}$$

(11) $$\begin{array}{c} \text{FOR}\cdot fIN\psi . \end{array}$$

(12) $$\begin{array}{c} {\text{IFF}}_{1}\left(m\left(G\cup \left\{f\right\}\right)\right)\geq \varepsilon . \end{array}$$

(13) $$\begin{array}{c} M=M\cup \left\{m\left(G\cup \left\{f\right\}\right)\right\}. \end{array}$$

(14) $$\begin{array}{c} f=\underset{f^{\prime }\in \psi }{\arg\max}F_{1}\left(m\left(G\cup \left\{f^{\prime }\right\}\right)\right). \end{array}$$

(15) $$\begin{array}{c} G=G\cup \left\{f\right\},\psi =\psi -\left\{f\right\}. \end{array}$$

(16) $$\begin{array}{c} \text{RETURNM}. \end{array}$$

For a given post, each model in the model set *M* is used to classify *P* (class label), and the most class label is used as the final tag of the post *P*. If the number of two kinds of labels is the same, the class label with the higher prior probability is selected as the final tag of *P* [14].

RETRACTED

In order to intuitively present the uncertainty of the analysis of the survey results, two horizontal axes were designed as one-dimensional projection spaces of two kinds of information fusion. After the survey objects were projected onto the projection axis, the same questionnaire was connected. The color of the projection point was determined by the average distance difference between the point and other points in different projection spaces. It shows that the uncertainty of the analysis results of the survey objects corresponding to this point is stronger, and further investigation and analysis are needed. Figures 2 and 3 show the visualization results of the uncertainty of multisource information fusion. Figures 2 and 3 show the projection results of different information fusion data in two-dimensional space, and the color mapping comes from the uncertainty measurement in one-dimensional projection space [15].

### 2.6. The Visual Analysis System of the Multisource Mental Health Questionnaire

In order to further facilitate experts in the field to quickly explore and comprehensively analyze the multisource college students' mental health information fusion data, this paper integrates the abovementioned data mining algorithm and visual design and realizes the visual analysis system tool. The interface is shown in Table 1 and Figures 4–6. It can be seen that the designed system is mainly composed of the visualization windows shown in Table 1 and Figures 4–6. Table 1 shows the overview of the original data and the specific information of students and answers to the questionnaire, including the type of questionnaire, the number of questions, and the answers information of specific interested students; Figure 4 shows the detailed information of the individual questionnaire of the object of interest, and the Circos diagram shows the specific answer information of the students specified by the user interaction; and Figures 5 and 6 show the correlation analysis interface. It supports users to select initial attributes interactively, draw attribute similarity paths with minimum cost, and parallel coordinates are arranged according to the path.

RETRACTED

## 3. Results and Analysis

In order to verify the effectiveness and practicability of the algorithm and system in this paper, we use the actual UPI and SCL-90 questionnaire data of 278 students at a certain university provided by the cooperation unit. This section will be mainly from the case analysis and user feedback analysis to verify [16].

### 3.1. Case Study

In the process of specific case analysis, users with experience and needs of mental health data analysis are invited to use the designed system to summarize, record, and analyze the user's data analysis process and feedback from the perspective of student individual situation analysis, survey angle correlation analysis, and information fusion uncertainty analysis.

#### 3.1.1. Analysis of Individual Health Status

Users hope that through the system comprehensive analysis and judgment of college students' individual mental health status, they will accurately understand the correlation between different attribute characteristics. The user randomly selected two students, and the specific visualization results of multisource information fusion are shown in Figures 7 and 8. The distribution of chord diagrams in Figure 7 is very dense, which indicates that student A is most likely to have mental health problems. In order to further determine the severity of the mental health problems of the respondents, the user moved the mouse over the inner ring and selected the topics of interest to understand the relevant situation. It was found that most of the score curves corresponding to student A were at a high level. It is concluded that the mental health problems of student A are more serious, and the symptoms of depression and schizophrenia are prominent. It is necessary to seek psychological experts for corresponding treatment. In contrast, student B's mental health problems are also more serious, and users judge that student B still needs further diagnosis and treatment [17]. Therefore, there are some differences between the two different questionnaires UPI and SCL-90, and the differences between the attributes need to be further analyzed according to the attributes. After the corresponding data analysis, the user feedback is as follows: the design of a multisource information fusion visualization scheme can help users quickly perceive the mental health status of the survey objects, and through simple interaction, it can effectively analyze and find the specific survey attributes of the survey objects with problems.

RETRACTED

#### 3.1.2. Attribute Correlation Analysis of the Multisource Questionnaire Survey

In order to further observe and analyze the attribute correlation of multisource information fusion, users carefully observe the attribute similarity distribution map and the results show that the attribute distribution distance in the same questionnaire survey system shown in Figure 9 is relatively close, while that of the same survey angle shown in Figure 10 is relatively close, except for most attributes related to mental factors. There were significant differences in the distribution of the two questionnaires related to the body. When users click on a point in the attribute similarity distribution map, the minimum cost path from this point is presented in the form of an animation line. At the same time, the order of parallel axes on the right side is optimized accordingly. Users click on different attributes of the multisource questionnaire in turn to observe the feature transformation. Figures 9–12 show the similarity distribution of two different attributes; that is, experts can find two kinds of attributes with obvious characteristics by clicking.  Figure 11 shows the minimum cost path and parallel axis sequencing drawn from the schizophrenia attribute of UPI [18]. It turns out that the higher the similarity, the higher the similarity of data line distribution between the attributes. The more obvious phenomenon is that the three symptoms with the highest correlation with UPI belong to UPI, and the symptom with the lowest correlation belongs to the somatization of SCL-90, which indicates that the correlation between schizophrenia symptoms and somatization is the lowest.  Figure 12 shows the attribute similarity distribution map and corresponding parallel coordinates drawn from the somatization symptoms of SCL-90. The three symptoms with high correlation also belong to the same questionnaire SCL-90, and the three symptoms with the lowest correlation belong to the distribution of similarity of different attributes of UPI [19]. According to users, in multisource questionnaires, such as UPI and SCL-90, different symptoms of the same questionnaire had a strong correlation, but different symptoms of different questionnaires had strong correlation, and the correlation was weak; different questionnaires have a high correlation with the design of the same symptom; in UPI and SCL-90, somatic symptoms had the lowest correlation with other symptoms; the results of the correlation analysis of the multisource questionnaire are similar to the actual situation. It has strong persuasion. Therefore, the multisource college students' mental health questionnaire has certain relevance and complementarity.

RETRACTED

#### 3.1.3. Visualization of Uncertainty of Multisource Survey Results

Due to the differences in the survey directions and angles of different questionnaires, it is often easy to lead to different analysis results, which will interfere with the comprehensive survey, collaborative analysis, and precise treatment of college students' mental health. Users select different individual students by clicking the dimensionality reduction point in Figure 13, and through further observation, the user found that the connection between the student's SCL-90 and UPI judgment results was gentle. In Figure 13, the student's dimensionality reduction points were scattered outside the whole, but in Figure 14, they were in a dense area, and there was a big difference between the two judgment results [20].

## 4. Conclusion

The MDS algorithm is used to reduce the dimension of SCL-90 and UPI data and project them into the low-dimensional space. The geometric space distance of the projection points indicates the differences among students. The differences of multisource questionnaire analysis results are effectively evaluated by the geometric space difference measurement, and the color mapping is used to effectively guide users to pay attention to students with uncertain analysis results. Effectively integrate users' prior knowledge to judge the mental health status of college students. A large number of visual analysis results and user feedback further verify the effectiveness and practicability of the visual analysis tool designed.

## Figures and Tables

**Figure 1:** Visualization result of multisource information fusion.

**Figure 2:** The Scl-90 projection multisource questionnaire uncertainty visualization results.

**Figure 3:** Visualization results of the uncertainty of UPI projection multisource questionnaire.

**Figure 4:** Multisource questionnaire fusion analysis.

**Figure 5:** Correlation analysis of the SCL-90 multisource survey.

**Figure 6:** Correlation analysis of the UPI multisource survey.

**Figure 7:** Comparative analysis of the visualization results of student A multisource questionnaire fusion.

RETRACTED

**Figure 8:** Comparative analysis of the visualization results of student B multisource questionnaire fusion.

**Figure 9:** Distribution of attribute characteristics of different questionnaires.

**Figure 10:** The onset of schizophrenia (UPD).

**Figure 11:** Distribution of mental and physical attributes.

**Figure 12:** Initiation of somatization (SCL-90).

**Figure 13:** Dimension reduction results of SCL-90 respondents.

**Figure 14:** UPI survey object dimension reduction results.

**Table 1:** Data overview and questionnaire basic information.

	Number of people	Raise the number	Efficiency
UPI	278	64	100
SCL-90	278	90	100

## Data Availability

The datasets used and/or analyzed during the current study are available from the author on reasonable request.
